# Dioscorea nipponica Makino Relieves Ovalbumin-Induced Asthma in Mice through Regulating RKIP-Mediated Raf-1/MEK/MAPK/ERK Signaling Pathway

This article has been retracted.

**DOI:** 10.1155/2022/8077058

**Published:** 2022-06-15

**Authors:** Weiyi Wang, Liying Xu, Lingming Zhou, Shanhong Wan, Libin Jiang

**Affiliations:** ^1^Department of Respiratory and Critical Care Medicine, The First Affiliated Hospital of Zhejiang Chinese Medical University (Zhejiang Provincial Hospital of Traditional Chinese Medicine), Hangzhou 310003, China; ^2^Department of Emergency, The First Affiliated Hospital of Zhejiang Chinese Medical University (Zhejiang Provincial Hospital of Traditional Chinese Medicine), Hangzhou 310003, China; ^3^Department of Respiratory Medicine, Zhejiang Chinese Medical University, Hangzhou 310053, China; ^4^Department of Geriatric Medicine, The First Affiliated Hospital of Zhejiang Chinese Medical University (Zhejiang Provincial Hospital of Traditional Chinese Medicine), Hangzhou 310003, China

## Abstract

**Purpose:**

Dioscorea nipponica Makino (DNM) is a traditional herb with multiple medicinal functions. This study is aimed at exploring the therapeutic effects of DNM on asthma and the underlying mechanisms involving RKIP-mediated MAPK signaling pathway.

**Methods:**

An ovalbumin-induced asthma model was established in mice, which was further administrated with DNM and/or locostatin (RKIP inhibitor). ELISA was performed to detect the serum titers of OVA-IgE and OVA-IgG1, bronchoalveolar lavage fluid (BALF) levels of inflammation-related biomarkers, and tissue levels of oxidative stress-related biomarkers. The expression of RKIP was measured by quantitative real-time PCR, Western blot, immunohistochemistry, and immunofluorescence. HE staining was used to observe the pathological morphology of lung tissues. The protein expression of MAPK pathway-related proteins was detected by Western blot.

**Results:**

Compared with the controls, the model mice exhibited significantly higher serum titers of OVA-IgE and OVA-IgG1, BALF levels of IL-6, IL-8, IL-13, TGF-*β*1, and MCP-1, tissue levels of MDA and ROS, lower BALF levels of IL-10 and IFN-*γ*, and tissue level of GSH. DNM relieved the allergic inflammatory response and oxidative stress in the model mice. DNM also recovered the downregulation of RKIP and the pathological injury of lung tissues in asthma mice. In addition, the Raf-1/MEK/MAPK/ERK pathway in the model mice was blocked by DNM. Silencing of RKIP by locostatin weakened the relieving effects of DNM on asthma through activating the Raf-1/MEK/MAPK/ERK pathway.

**Conclusion:**

DNM relieves asthma via blocking the Raf-1/MEK/MAPK/ERK pathway that mediated by RKIP upregulation.

## 1. Introduction

Asthma is a respiratory disease characterized by airway inflammation and hyperresponsiveness [1]. Asthma is mostly occurred in childhood at a prevalence of 495 per 100,000 in comparison to that in adults at 92 per 100,000, which will affect about 400 million people worldwide by 2025 [2–4]. In clinical, asthma is accompanied by nonspecific symptoms, including recurrent wheeze, shortness of breath, cough, and variable expiratory airflow limitation [5]. To avoid symptom burden and exacerbation risk, anti-inflammation and bronchodilation are dominant for the treatment of asthma [6]. Inhaled corticosteroids (ICS) and bronchodilators are the most commonly used drugs for asthma; nevertheless, the responsiveness varies among individuals [7]. The discovery of more effective drugs against asthma without side effect is still needed.

In China, there is a long-term history of traditional Chinese medicine (TCM) use in the treatment of respiratory diseases including asthma [8]. A diversity of TCMs have been determined to have therapeutic potential for asthma, such as Cordyceps sinensis [9], Astragalus membranaceus [10], Carthamus tinctorius [11], Atractylodis rhizome [12], and Cimicifugae Rhizoma [13]. Dioscorea nipponica Makino (DNM) is a perennial twining herb that exhibits a variety of medicinal functions, such as anti-inflammation, antitussive, antitumor, antipain, panting-calming and phlegm-dispelling, immune regulation, and cardiovascular system protection [14]. DNM has been widely used to protect against rheumatoid arthritis, Kashin-Beck disease, sprains, bruises, bronchitis, and cough in China [14, 15]. It is noted that DNM may also contribute to the remission of asthma. Ou-Yang et al. concluded the pharmacological profile of DNM and demonstrated that DNM possesses the favorable antiasthmatic effect that was validated in mice with asthma [14]. Junchao et al. have shown that diosgenin from DNM inhibits the inflammation in asthmatic mice [16]. Wang et al. have found that saponins from DNM mitigate the effects of IL-17A on the proliferation, migration, and cytoskeleton remodeling of human airway smooth muscle cells in vitro, indicating a candidate for treating asthma-associated airway hyperresponsiveness [17]. However, the specific effects of DNM and the underlying molecular mechanisms in asthma have not been fully revealed.

MAPK signaling pathway is a convergent node responses to diverse stimulus, such as metabolic stress, DNA damage, protein dysregulation, external growth factor signaling, cell-matrix interaction, and cell-cell communication [18]. By regulating the transcription of target genes, MAPK pathway plays a critical role in fundamental cellular functions (cell proliferation, apoptosis, differentiation, and migration), tumorigenesis, extrinsic stress response, and metabolic reprogramming [19–21]. Notably, MAPK pathway is also the action target of many TCMs against asthma. For example, hydroxysafflor yellow A attenuates airway resistance, inflammation, and pathologic changes of OVA-induced asthma in guinea pigs through inhibiting the MAPK pathway [11]. Icariin alleviates pulmonary inflammation, airway remodeling, and the proliferation of airway smooth muscle cells through inhibiting the MAPK/ERK pathway in a mouse model of OVA-induced asthma [22]. Ginkgolide B inhibits OVA-induced eosinophilia in lung tissues and mucus hypersecretion in the airway in a mouse model [23]. In addition, previous studies have also determined that DNM exhibits a great potential in the treatment of gouty arthritis via regulating MAPK pathway [24, 25]. However, the action mechanisms of DNM in asthma involving the MAPK pathway are not entirely understood.

In this study, the therapeutic potential of DNM was analyzed in a mouse model of ovalbumin- (OVA-) induced asthma. The action mechanisms of GNV involving RKIP-mediated MAPK signaling pathway were further determined. The objective of this study is to investigate the therapeutic efficacy and mechanism of DNM on asthma, thereby providing promising natural drug and target therapeutic strategy for asthma treatment.

## 2. Methods

### 2.1. Model Establishment and Grouping

Animal experiments were approved by the ethical committee of The First Affiliated Hospital of Zhejiang Chinese Medical University. Female BALB/c mice (HFK Bio, Beijing, China) at 8 weeks old were used to establish OVA-induced asthma model as previously described [26]. All mice were raised in a laboratory room with 24 ± 2°C, 60 ± 5% humidity, and 12 h light/dark cycle. Simply, mice were sensitized by intraperitoneal injection of 200 *μ*L OVA inducer (50 *μ*g OVA and 0.8 mg aluminum hydroxide dissolved in 0.9% physiological saline; Sigma-Aldrich, MO, USA) for twice with an interval of 14 days (days 1 and 14). After injection, mice were exposed to 2% OVA (dissolved in 3 mL 0.9% physiological saline) for 20 min every 3-4 days (days 14, 17, 20, 23, and 27). DNM (a natural herb) with an active ingredient of Dioscin (0.2505 ± 0.0003 ng/uL, 3.074 ± 0.053%, HPLC) was purchased from Tongrentang (Beijing, China). The OVA-sensitized and OVA-challenged mice (model mice) were randomly divided into 5 groups (*N* = 6 each group) and received different administrations for 14 days following OVA injection. Model group: it is a group of model mice without administration; model+DNM: model mice were orally administrated with 1.95 g/kg DNM; model+locostatin (RKIP inhibitor; Darmstadt, Germany): model mice were intraperitoneally injected with 0.5 mg/kg locostatin; model+DNM+locostatin: model mice were orally administrated with 1.95 g/kg DNM and intraperitoneally injected with 0.5 mg/kg locostatin; model+prednisone acetate (PA): model mice were gavaged with 5 mg/kg PA. Normal mice without OVA injection and oral administrated with physiological saline were used as the control group (*N* = 6). After the last intervention (day 27), mice were anaesthetized with sodium pentobarbital (50 mg/kg, intraperitoneal injection) and sacrificed by cervical dislocation.

### 2.2. Enzyme-Linked Immunosorbent Assay (ELISA)

The blood samples were collected from mice via the retroorbital plexus. The serum titers of OVA-IgE and OVA-IgG1 were measured using commercial ELISA kits (Mlbio, Shanghai, China). The bronchoalveolar lavage fluid (BALF) was collected by 3 times of intratracheal instillation with PBS, and the supernatants were used for detecting inflammation-related biomarkers, including the IL-6, IL-8, IL-10, IL-13, IFN-*γ*, TGF-*β*1, and MCP-1. In addition, the resected lung tissues were collected for measuring the contents of GSH, MDA, and ROS. The above parameters were all measured using corresponding commercial ELISA kits in accordance with the manufacturer's instructions (IL-6/IL-8/IL-10/IL-13/IFN-*γ*, Mlbio; TGF*β*1/MCP-1, Thermo Fisher Scientific, CA, USA; GSH, Jiancheng, Nanjing, China; MDA, Solarbio, Beijing, China; and ROS, QualitYard, Beijing, China). The levels of related parameters were finally calculated according to established standard curves.

### 2.3. Quantitative Real-Time PCR (qRT-PCR)

Total RNAs were extracted from lung tissues using TRIZOL reagent (Invitrogen, Carlsbad, CA, USA). By using the template of cDNAs that reversely transcribed by FastKing First-strand cDNA Synthesis Mix (Tiangen, Beijing, China), qRT-PCR was performed on MX3000P Real-Time PCR instrument (Agilent, Santa Clara, CA, USA). The qRT-PCR program was an initial 95°C for 3 min and 40 cycles of 95°C for 15 s and 62°C for 40 s. The relative expression of RKIP was calculated by the 2^-∆∆Ct^ method. GAPDH was used as the internal control. The primers used in qRT-PCR are listed in Table 1.

### 2.4. Hematoxylin-Eosin (HE) Staining

The resected lung tissues were fixed with 4% formalin for 24 h, embedded in paraffin, and sectioned into 5 *μ*m. After dewaxing, the sections were stained with hematoxylin for 5 min and then with eosin for 1 min. The stained sections were finally observed under an optical microscope (Olympus, Japan).

### 2.5. Immunohistochemistry (IHC) and Immunofluorescence (IF)

The paraffin sections of lung tissues were further used in IHC and IF for detecting the expression of RKIP. After dewaxing, the sections were microwave irradiated in citrate buffer for 15 min at 95°C, soaked in 3% H_2_O_2_ for 20 min, blocked with 5% goat serum for 15 min, and incubated with anti-RKIP (1 : 100, Abcam) for 12 h at 4°C. Then, the sections received 1 h of incubation with HRP-IgG (1 : 500, Abcam) for IHC and with Alexa Fluor® 488-IgG for IF (1 : 500, Abcam) at 25°C. Sections used in IHC were visualized with diaminobenzidine and observed under an optical microscope (Olympus). Sections used in IF were counterstained with DAPI and observed under a confocal microscope (ULTRAVIEW VOX, Perkin Elmer, USA).

### 2.6. Western Blot

The protein samples were isolated from lung tissues by lysing in RIPA buffer (Beyotime) and quantified using BCA Protein Assay Kit (Beyotime). The proteins were separated by 10% SDS-PAGE and then transferred onto PVDF membranes. After blocked with 5% nonfat milk for 1 h, the membranes were incubated with primary antibodies (anti-RKIP (ab76582) and anti-GAPDH (ab181602), Abcam, 1 : 1,000; anti-(p)-Raf-1 (Cat# AP3922a) and -(p)-ERK1/2 (Cat#AP3906a), Abcepta, 1 : 1,000; and anti-(p)-MEK1/2 (#9154S), -(p)-p38 MAPK (#4511), Cell Signaling Technology; 1 : 1,000) at 4°C overnight. Subsequently, the membranes were further incubated with secondary antibody (HRP, 1 : 5,000, ab205718, Abcam) for 1 h at 25°C. The protein bands were visualized using an ECL kit (Thermo Fisher Scientific, CA, USA) and quantified by ChemiDoc imaging system (Bio-Rad, CA, USA). GAPDH served as an internal control.

### 2.7. Statistical Analysis

Statistical analysis was performed using the software of GraphPad Prism 7. All data were expressed as the mean ± standard deviation. Comparisons among different groups were determined by one-way analysis of variance (ANOVA) followed by Tukey's test. A *P* value less than 0.05 represented significantly different.

## 3. Results

### 3.1. DNM Relieves the Allergic Response in Asthma Mice through Upregulating RKIP

To reveal the effects of DNM in asthma, a mouse model of OVA-induced asthma was established. As shown in Figures 1(a) and 1(b), the serum titers of OVA-IgE and OVA-IgG1 were both significantly higher in the model mice than those in the controls (*P* < 0.001). qRT-PCR showed that the mRNA expression of RKIP was significantly decreased in the model mice compared with the controls (*P* < 0.001, Figure 1(c)). In consistent with PA, DNM significantly decreased the serum titers of OVA-IgE and OVA-IgG1 and increased RKIP expression in the model mice (*P* < 0.001, Figures 1(a) and 1(c)). RKIP was then silenced by locostatin to determine the action mechanisms of DNM relating with RKIP. The results showed that the intervention of locostatin increased the serum titers of OVA-IgE and OVA-IgG1 and downregulated RKIP in the model mice (*P* < 0.05, Figures 1(a) and 1(c)). In addition, locostatin weakened the inhibitory effects of DNM on the allergic response of asthma via downregulating RKIP (*P* < 0.05, Figures 1(a) and 1(c)). In consistent with the mRNA expression of RKIP, constant changes were also determined on the protein expression of RKIP in lung tissues by IHC and IF (Figures 2(a) and 2(b)).

### 3.2. DNM Relieves the Inflammatory Response in Asthma Mice through Upregulating RKIP

Since asthma is a chronic inflammatory disease, some inflammation-related biomarkers were detected in the BALF. As shown in Figures 3(a)–3(e), the BALF levels of IL-6, IL-8, IL-13, TGF-*β*1, and MCP-1 were significantly higher in the model mice than those in the controls (*P* < 0.001). On the contrary, significantly lower levels of IL-10 and IFN-*γ* were revealed in BALF of the model mice compared with the controls (*P* < 0.001, Figures 3(f) and 3(g)). The intervention of DNM significantly decreased the IL-6, IL-8, IL-13, TGF-*β*1, and MCP-1 levels and increased the IL-10 and IFN-*γ* levels in BALF of the model mice (*P* < 0.01). Consistent results with DNM were observed in a positive drug PA in the model mice (*P* < 0.01). In addition, locostatin showed opposite effects on the above biomarkers with the DNM via inhibiting RKIP (*P* < 0.01). Notably, locostatin weakened the effects of DNM on reducing IL-6, IL-8, IL-13, TGF-*β*1, and MCP-1 and on elevating IL-10 and IFN-*γ* in BALF of the model mice (*P* < 0.05, Figures 3(a)–3(g)).

### 3.3. DNM Relieves the Oxidative Stress in Asthma Mice through Upregulating RKIP

Oxidative stress is closely associated the asthmatic inflammation and severity. Here, ELISA determined significantly higher contents of MDA and ROS and lower content of GSH in lung tissues of the model mice compared with the controls (*P* < 0.001). Both DNM and PA could decrease the MDA and ROS contents and increase the GSH content in the model mice (*P* < 0.01). Via inhibiting RKIP, locostatin presented contrary effects on the above biomarkers with DNM (*P* < 0.01). In addition, locostatin weakened the effects of DNM on decreasing MDA and ROS and on increasing GSH in lung tissues of the model mice (*P* < 0.05, Figures 3(h)–3(j)).

### 3.4. DNM Relieves the Pathological Injury of Lung Tissues in Asthma Mice through Upregulating RKIP

The pathological morphology of lung tissues was observed by HE staining. As shown in Figure 4, normal mice (control group) exhibited clear alveolar texture, regular bronchial lumen, intact airway mucosal epithelium and alveolar wall, and no inflammatory cell infiltration. However, obvious pathological injury was observed in lung tissues of the model mice, presenting bronchial lumen stenosis, capillary edema, partial alveolar fusion, airway epithelium abscission, and massive inflammatory cell infiltration. The pathological injury in the model mice was relieved by DNM or PA but was aggravated by locostatin to some degrees. Locostatin also weakened the relieving effects of DNM on the pathological injury of lung tissue in the model mice (Figure 4).

### 3.5. DNM Blocks the Raf-1/MEK/MAPK/ERK Signaling Pathway in Asthma Mice through Upregulating RKIP

Because RKIP is involved in the inhibition of the MAPK signaling pathway by mediating Raf-1, the action mechanisms of DNM involving the Raf-1/MEK/MAPK/ERK pathway were further analyzed. As shown in Figure 5, the protein expression of p-Raf-1, p-MEK1/2, p-p38 MAPK, and p-ERK1/2 was significantly higher in the model mice than that in the controls (*P* < 0.001). In consistent with PA, DNM inhibited the activation of the Raf-1/MEK/MAPK/ERK pathway in the model mice (*P* < 0.001). In addition, locostatin-induced inhibition of RKIP further enhanced the activation of the Raf-1/MEK/MAPK/ERK pathway in the model mice, evidenced by upregulated p-Raf-1, p-MEK1/2, p-p38 MAPK, and p-ERK1/2 (*P* < 0.05). Locostatin also reversed DNM-induced inhibition of the Raf-1/MEK/MAPK/ERK pathway (*P* < 0.05).

## 4. Discussion

Asthma is an inflammatory condition of the respiratory tract that driven by T-helper 2- (Th2-) immune response [27]. So far, a variety of TCMs have been widely used for the treatment of asthma, including the DNM. However, fundamental researches on the function and underlying molecular mechanisms of DNM in asthma are limited. In this study, an OVA-induced asthma was established in mice to determine the role of DNM. Firstly, we found that DNM significantly decreased the serum titers of OVA-IgE and OVA-IgG1 in the asthma mice. IgE and IgG are known to be central in the immunopathogenesis of allergic asthma, which are positively associated with the phenotypes of bronchial airway inflammation and hyperreactivity and eosinophil enrichment [28–30]. Our findings indicate that the intervention of DNM inhibited the allergic response of asthma mice against OVA. In addition to the increased immunoglobulins, asthma is also characterized by increased Th2 type cytokines [31]. IL-13 is one of the most important Th2-type cytokines that exerts a critical role in eosinophilic inflammation, mucus hypersecretion, airway hyperactivity, and airway remodeling [32]. In this study, DNM-induced decreasing of IL-13 level in BALF of model mice illustrates that DNM is able to inhibit Th2-type response in asthma. In addition, DNM also significantly decreased IL-6, IL-8, MCP-1, and TGF-*β*1 and increased IL-10 and IFN-*γ* in BALF of the model mice. These results further indicate that the intervention of DNM inhibited the allergic inflammatory response in asthma. On the other hand, oxidative stress is also involved in asthmatic inflammation and severity, and targeting oxidizing molecules combined with inflammatory mediators has become a novel therapeutic strategy for asthma [33, 34]. In this study, the MDA and ROS levels were decreased and the GSH level was increased by DNM in lung tissues of asthma mice. These findings indicate that DNM may be benefit for the treatment of asthma through inhibiting oxidative stress. Furthermore, the HE staining directly confirmed the alleviating effect of DNM on asthma, evidenced by a mild pathological injury in lung tissues of the model mice.

Furthermore, the potential molecular mechanism by which DNM exerts the therapeutic effect on asthma was investigated. RKIP, a member of the phosphatidylethanolamine-binding protein family, is a pivotal modulator in the inflammatory and immune system via interacting with multiple signaling molecules [35, 36]. It has been reported that RKIP plays a substantial role in asthma via interacting with diverse functional proteins, such as Raf-1, MUC5AC, GRK2, and 15LO1 [37]. Therefore, RKIP is a promising target for the therapeutic intervention of DNM on asthma. In this study, a downregulated RKIP was observed in OVA-induced asthma mice. This result is consistent with a previous study that the expression of RKIP was decreased in the peripheral blood of patients with asthma [38]. Lin et al. have also revealed that the RKIP deficiency in mast cells render mice more sensitive to IgE-Fc*ε*RI-mediated allergic response and OVA-induced airway inflammation [38]. Our findings showed that DNM significantly increased the expression of RKIP in OVA-induced asthma mice. We suspect that the upregulation of RKIP may contribute to the alleviating effect of DNM in asthma. Our subsequent results further determined this hypothesis, evidenced by that the inhibition of RKIP by locostatin weakened the relieving effects of DNM on the allergic inflammatory response, oxidative stress, and pathological injury in asthma mice.

The function of RKIP is inseparable from its interaction with multiple signaling molecules involving inflammatory processes [37]. Under homeostatic condition, RKIP appears to exhibit anti-inflammatory role through inhibiting the ERK/MAPK pathways [37]. Evidence has proved that RKIP can inhibit Raf-1-mediated activation of the MAPK/ERK signaling pathway by suppressing the phosphorylation of Raf-1 [39]. Consistently, we found that the inhibition of RKIP by locostatin enhanced the activation of the Raf-1/MEK/MAPK/ERK pathway in asthma mice. MAPK pathway is a classical inflammatory pathway that involved in the pathology of diverse human inflammatory diseases, including cancer, neurodegenerative disorders, diabetes, cardiovascular diseases, and inflammatory bowel diseases [40]. There many potential drugs have been determined to treat asthma through inhibiting the MAPK pathway, such as hydroxysafflor yellow A [11], icariin [22], ginkgolide B [23], caffeic acid phenethyl ester [41], dehydrodieugenol [42], and paeonol [43]. In this study, the activated Raf-1/MEK/MAPK/ERK pathway in asthma mice was also inhibited by DNM, indicating a potential action mechanism of DNM. Zhou et al. have shown that the saponin fraction from DNM exerts anti-inflammation effects on gouty arthritis by inhibiting MAPK pathway [24]. To combine with the promoting role of DNM on RKIP, we suspect that DNM may upregulate RKIP to block the Raf-1/MEK/MAPK/ERK pathway, thereby alleviating asthma.

## 5. Conclusion

In conclusion, DNM relieves OVA-induced asthma in a mouse model, evidenced by decreased allergic inflammatory response, oxidative stress, and pathological injury of lung tissues. In addition, DNM blocks the Raf-1/MEK/MAPK/ERK pathway through upregulating RKIP, presenting an underlying action mechanism of DNM against asthma. This study provides a promising natural drug with low side effects for the treatment of asthma. Meanwhile, the molecular mechanism of DNM treating asthma was revealed, which provides new guidance for the target therapy of asthma. However, this study is limited by the unclear bioactive components in DNM. Further, we can explore the potential bioactive components of DNM against asthma, which may exert the better therapeutic efficacy on asthma. Thus, other potential molecular mechanisms of DNM against asthma can be deciphered based on bioactive compounds. In-depth researches on the action mechanisms of DNM in asthma are also needed.

## Figures and Tables

**Figure 1:** DNM inhibits the allergic response via downregulating RKIP in a mouse model of OVA-induced asthma. (a) Serum titers of OVA-IgE; (b) serum titers of OVA-IgG1; (c) the mRNA expression of RKIP. ^∗∗∗^*P* < 0.001 vs. control; ^#^*P* < 0.05, ^##^*P* < 0.01, and ^###^*P* < 0.001 vs. model; ^&&^*P* < 0.01 and ^&&&^*P* < 0.001 vs. model+DNM. ELISA and qRT-PCR were performed in triplicate in six independent mice.

**Figure 2:** The protein expression of RKIP in lung tissues of OVA-induced asthma mice. (a) IHC; (b) IF. IHC and IF were performed in six independent mice.

**Figure 3:** DNM inhibits the allergic inflammatory response and oxidative stress via downregulating RKIP in a mouse model of OVA-induced asthma. (a) IL-6 in BALF; (b) IL-8 in BALF; (c) IL-13 in BALF; (d) TGF-*β*1 in BALF; (e) MCP-1 in BALF; (f) IL-10 in BALF; (g) IFN-*γ* in BALF; (h) MDA in lung tissues; (i) ROS in lung tissues; (j) GSH in lung tissues. ^∗∗∗^*P* < 0.001 vs. control; ^#^*P* < 0.05, ^##^*P* < 0.01, and ^###^*P* < 0.001 vs. model; ^&^*P* < 0.05, ^&&^*P* < 0.01, and ^&&&^*P* < 0.001 vs. model+DNM. ELISA was performed in triplicate in six independent mice.

**Figure 4:** The pathological morphology of lung tissues in a mouse model of OVA-induced asthma was assessed by HE staining. HE was performed in six independent mice.

**Figure 5:** The activation of the Raf-1/MEK/MAPK/ERK signaling pathway in mice with OVA-induced asthma was detected by Western blot. Western blot was performed in six independent mice. ^∗∗∗^*P* < 0.001 vs. control; ^#^*P* < 0.05, ^##^*P* < 0.01, and ^###^*P* < 0.001 vs. model; ^&^*P* < 0.05, ^&&^*P* < 0.01, and ^&&&^*P* < 0.001 vs. model+DNM.

**Table 1:** Primer sequences for qRT-PCR.

Gene	Species	Forward primer (5′-3′)	Reverse primer (5′-3′)
RKIP	Mice	AGGTTATGAACAGGCCCAGC	AGACATAGCGGTGGAGACCT
GAPDH	Mice	TGTGGGCATCAATGGATTTGG	ACACCATGTATTCCGGGTCAAT

## Data Availability

The data used to support the findings of this study are available from the corresponding author upon request.

## Additional Points

*Highlight*. (1) DNM alleviates the allergic response in asthma mice. (2) DNM relieves the inflammation and oxidative stress in asthma mice. (3) GNV relieves the pathological injury of lung tissues in asthma mice. (4) GNV upregulated RKIP and blocked Raf-1/MEK/MAPK/ERK pathway
